RETRACTED

# Influence of miR-1 on Nerve Cell Apoptosis in Rats with Cerebral Stroke via Regulating ERK Signaling Pathway

**DOI:** 10.1155/2021/9988534

**Published:** 2021-08-19

**Authors:** Yuanding Jiang, Tao Wang, Jian He, Quan Liao, Jingjing Wang

**Affiliations:** ^1^Department of Neurosurgery, The Second Affiliated Hospital of South China University, Hengyang, 421001 Hunan Province, China; ^2^Department of Hemodialyses Room, The Second Affiliated Hospital of South China University, Hengyang, 421001 Hunan Province, China

## Abstract

To explore the effect of miR-1 on neuronal apoptosis in rats with stroke through the ERK signaling pathway. *Methods*. Forty male rats (180-220 g) were selected and randomly divided into the sham, model, miR-1 inhibitor, and miR-1 mimic groups (10 rats per group) by average body weight. Cerebral ischemia/reperfusion (I/R) models were established using a modified middle cerebral artery wire thrombosis (MCAO) method in rats in the model group, miR-1 inhibitor group, and miR-1 mimic group. After the successful model establishment, the miR-1inhibitor group and miR-1 mimic group were intravenously injected with miR-1 inhibitor and miR-1 mimic, respectively, once a day for 3 days. The sham and model groups were given the same dose of normal saline. TTC staining was applied to detect the cerebral infarct size and calculate the infarct volume. Histopathological changes in the hippocampus of rat brains were observed by HE staining. Flow cytometry was used to detect neuronal apoptosis in rat brains. The mRNA expressions of miR-1, ERK1/2, Bcl-2, and Bax in rat brain tissues were determined by QRT PCR, and the protein levels of ERK1/2, Bcl-2, Bax, and caspase-3 were determined by Western blot analysis. *Results*. Compared with the sham group, the neurological impairment score, cerebral infarct size, and volume of rats in the model group were significantly increased (*p* < 0.05). Compared with the model group, the neurological impairment score, cerebral infarct size, and volume were significantly increased in the miR-1 mimic group and significantly decreased in the miR-1 inhibitor group (*p* < 0.05). In the model group, the hippocampal tissue of rats had malaligned cells, neuron cell atrophy became smaller, the intercellular spaces became larger, and vacuoles appeared. Compared with the model group, the miR-1 inhibitor group could effectively alleviate the pathological changes in the hippocampus, and the miR-1 mimic group could significantly add to the pathological changes in the rat hippocampus. Compared with the sham group, the mRNA expression of miR-1 and Bax in the brain of model rats increased significantly (*p* < 0.05), and the mRNA expression of ERK1/2 decreased significantly; Compared with the model group, the miR-1 and Bax mRNA expressions in the brain tissues of rats in the miR-1 inhibitor group were significantly decreased, the ERK1/2 and bcl-2 mRNA expressions were significantly increased, and the miR-1 and Bax mRNA expressions in the brain tissues of rats in the miR-1 inhibitor group were significantly decreased, and the Bcl-2 mRNA expression was significantly increased (*p* < 0.05). Compared with the sham group, neuronal apoptosis was increased in the brain tissues of rats in the model group and miR-1 mimic group. Compared with the model group, neuronal apoptosis was decreased in the brain tissues of rats in the miR-1 inhibitor group. Compared with the sham group, the ERK1/2 proteins in the model group were significantly decreased, the Bcl-2, Bax, and caspase-3 proteins were significantly increased, and the ERK1/2, Bcl-2, Bax, and caspase-3 proteins in the miR-1 inhibitor group and miR-1 mimic group were significantly increased. Compared with the model group, the protein levels of ERK1/2 and Bcl-2 in the miR-1 inhibitor group were significantly increased, the proteins of Bax and caspase-3 were significantly decreased, and the protein levels of ERK1/2 and Bcl-2 in the miR-1 inhibitor group were significantly increased (*p* < 0.05). *Conclusions*. miR-1 can interfere with neuronal apoptosis in rats with stroke through the ERK signaling pathway.

RETRACTED

## 1. Introduction

Cerebral stroke, also known as cerebralvascular accident, is a kind of acute and sudden cerebrovascular disease. It is caused by obstruction and rupture of cerebral vessels, leading to blood stasis, preventing the blood from entering the brain, and triggering related diseases to hypoxic injury in the brain tissues, including ischemic stroke and hemorrhagic stroke [1]. Clinically, ischemic stroke is a common type of cerebral stroke, which may be induced by carotid artery stenosis and vertebral artery occlusion, mostly in males aged over 40 years old, and can result in death in severe cases. The mortality rate of hemorrhagic stroke of the patients with cerebral stroke is much higher than that of ischemic stroke, according to studies. Besides, cerebral stroke is the main reason of disability among adults in China, seriously threatening the life and health of human [2–4]. However, there is no efficacious therapeutic measure in clinic at present.

Microribonucleic acids (miRNAs or miRs) are endogenous single-stranded noncoding small RNA molecules with 22 nucleotides in length [5]. They regulate the expression of their complementary messenger RNAs (mRNAs) at the posttranscriptional level, thus affecting multiple physiological and pathological processes such as neurogenesis, neuronal maturation, and development and regeneration of the nervous system [6]. Previous studies have shown that miR-1 is involved in the initiation and progression of several diseases, such as nerve injury [7–9], and the expression changes of miRNAs are time dependent after peripheral nerve injury.

RETRACTED

Although cerebral stroke is correlated with various factors in the body, studies related to the effect of miR-1 on neuronal apoptosis in rats with cerebral stroke are rarely reported. Currently, the exact mechanism of cerebral stroke in damaging the nerves remains unclear. Therefore, this research is aimed at exploring the influence of the extracellular signal-regulated kinase (ERK) signaling pathway on nerve cell apoptosis in rats with cerebral stroke by intervening in miR-1, providing certain experimental bases for the treatment of nerve cell apoptosis induced by cerebral stroke.

## 2. Materials and Methods

### 2.1. Laboratory Animals, Main Reagents, and Instruments

A total of 40 healthy male Sprague-Dawley rats aged 10-12 weeks old and weighing 180-220 g were selected and then divided into the sham-operation group (sham group, *n* = 10), model group (MCAO group, *n* = 10), miR-1 inhibitor group (*n* = 10), and miR-1 mimic group (*n* = 10) based on the average body weight. The cerebral ischemia/reperfusion (I/R) injury model was established as per the modified MCAO method [10]. Specifically, the rats were anesthetized by intraperitoneal injection of 20% urethane (5 mL/kg), fixed on an operation table, and disinfected. Then, the skin was cut open along the left neck, and the arteries were bluntly dissected. The external carotid artery was ligated, and the common carotid artery was clipped using an artery clamp. Later, an oblique incision was made at the external carotid artery, from which a specialized nylon suture (0.26 mm in diameter) for cerebral embolism was gently pushed in and stopped when feeling resistance. After that, the suture was tightened at the external carotid artery, and the incision was sutured and disinfected. 2 h later, the suture was pulled out. The body temperature of the rats was maintained at 37 ± 0.5°C during the whole surgical procedure.

In the sham group, all the operations were the same except for the operation of nylon suture for cerebral embolism. Criteria of successful modeling are as follows: The rats were scored using the EZ Longa method at 2 h after resuscitation [6]. The rats with a score of 1-3 points were selected as the objects of this research and randomly assigned into the MCAO group, miR-1 inhibitor group, and miR-1 mimic group, with 10 rats in each group, after the model was prepared successfully. In addition, 10 rats were set as the sham group. Subsequently, the rats in the miR-1 inhibitor group and miR-1 mimic group were intravenously injected with the miR-1 inhibitor and miR-1 mimic, respectively, once a day for 3 days in total, while those in the sham group and MCAO group were given an equal dose of normal saline (Table 1).

RETRACTED

The miR-1 inhibitor and miR-1 mimic were synthesized by Guangzhou Ribio Biotech Co., Ltd., and eosin staining solution was provided by Shenyang Chemical Reagent No. 5 Factory. Fluorescence quantitative polymerase chain reaction (qPCR) reagent and consumables were purchased from TaKaRa (Dalian, China), and goat anti-rabbit IgG primary antibodies (Abcam, Germany) and rabbit anti-rat horseradish peroxidase- (HRP-) labeled secondary antibodies (TIANGEN Biotech, China) were used for Western blotting. In addition, miRNeasy Mini kit (TIANGEN Biotech, China), PCR instrument (Thermo, USA), Gaoke TD-5A table-top low-speed centrifuge (Jintan Changzhou Instrument Factory, China), ultra-micro spectrophotometer (Thermo, USA), TGL-16G centrifuge (Shanghai Anting Scientific Instrument Factory, China), PT-3502B microplate reader (Thermo, USA), ECL instrument (Thermo, USA), and HH-4 digital thermostatic water bath (Changzhou City Jintan Huate Experimental Instrument Co., Ltd., China) were applied.

### 2.2. Methods

#### 2.2.1. 2,3,5-Triphenyltetrazolium Chloride (TTC) Staining Methods

The brain tissues of the rats were taken after the last drug administration, which were frozen at -20°C for 25 min and sliced to prepare frozen sections. Then, the sections were placed in 1% TTC solution, incubated at 37°C for 15 min, and fixed with 10% formaldehyde solution. Finally, the infarction area in the sections was measured using Image-Pro Plus software, so as to calculate the cerebral infarction volume. The red parts stand for noninfarcted tissues and the white parts for infarcted tissues.

#### 2.2.2. Fluorescence qPCR

The brain tissue samples stored in liquid nitrogen were taken out to extract the total RNA using a TRIzol reagent method, which was reversely transcribed according to the instructions of reverse transcription (RT) kit. Then, target genes were amplified as per the instructions of the qRT-PCR kit, with the RT product (complementary deoxyribonucleic acid (cDNA)) as the template. Fluorescence qPCR system: 10 *μ*L of qPCR Master Mix (2×), 1 *μ*L of PCR reverse primer, 2 *μ*L of cDNA, and 11 *μ*L of ddH_2_O. Finally, the results were calculated via 2^-△△Ct^ method (Table 2).

#### 2.2.3. Hematoxylin-Eosin (HE) Staining

The brain tissues fixed for 24 h were taken out, washed in clear water, and dehydrated with ethanol, followed by embedding in paraffin and slicing into sections. Then, the sections were stained with hematoxylin at room temperature for 10 min, washed with clear water for 30 min, and soaked in 1% hydrochloric acid for 30 s. After washing in clear water again for 30 s, the sections were stained with eosin at room temperature for 5 min, dehydrated with ethanol, and then sealed in neutral gel in ventilation environment. Finally, the changes in the brain tissues were observed under a microscope.

RETRACTED

#### 2.2.4. Detection of Cell Apoptosis via Flow Cytometry

Fresh brain tissues in each group were put in plates, added with normal saline, and cut into pieces using scissors, followed by homogenization in a tissue homogenizer. Then, the homogenate was aspirated and filtered into 10 mL centrifuge tubes by 100-mesh nylon nets, followed by centrifugation at 1000 rpm for 5 min and washing with normal saline for 3 times. Next, the cells were resuspended in 5 mL of PBS, filtered by 300-mesh nylon nets, and detected using a flow cytometer.

#### 2.2.5. Western Blot

*(1) Western Blotting*. The brain tissues of the rats taken out from liquid nitrogen were added with RIPA lysis buffer containing PMSF and homogenized in a glass homogenizer for 4 min. Later, the homogenate was collected and centrifuged at 12,000 rpm for 10 min. The supernatant was taken, mixed with 5× protein loading buffer and boiled for 3 min. After SDS-PAGE, the samples were transferred onto a polyvinylidene fluoride (PVDF) membrane. Subsequently, the PVDF membrane was sealed in 5% skim milk powder solution at room temperature for 1 h, incubated with correspondingly diluted antibodies (1 : 1000) at 4°C overnight, and washed with TBST for 5 min 3 times. Next, the membrane was sealed with relevant HRP-labeled antibodies (diluted at 1 : 5000) at 37°C for 1 h, followed by color development with developer and quantitative analysis using Quantity One software.

### 2.3. Data Analysis

The experimental data were analyzed via SPSS 19.0 software. The mean ± standard deviation ($\bar{\chi }\pm s$) was adopted for intragroup comparison, one-way analysis of variance was utilized for intergroup comparison, and *p* < 0.05 suggested statistical differences.

## 3. Results

### 3.1. Comparison of Neurological Deficit Score among Groups

As shown in Table 3, compared with the sham group, the neurological impairment scores of rats in the model group were significantly increased (*p* < 0.05). Compared with the model group, the neurological impairment scores of the miR-1 mimic group were significantly increased, as were the scores of the rats in the miR-1 inhibitor group (*p* < 0.05).

### 3.2. Comparison of Infarction Volume in Brain Tissues among Groups

As shown in Figure 1 and Table 4, compared with the sham group, the cerebral infarct size and volume of the model rats were significantly increased (*p* < 0.05).Compared with the model group, the cerebral infarct size and volume were significantly increased in the miR-1 mimic group, and the neurologic impairment score and the cerebral infarct size and volume were significantly decreased in the miR-1 inhibitor group (*p* < 0.05).

RETRACTED

### 3.3. Comparison of Pathological Changes in Hippocampal Tissues among Groups

In contrast with those in the sham group, the cells in the hippocampal tissues of the rats were arranged irregularly, the neuronal cells became atrophic and small, the intercellular space was increased, and vacuoles occurred in MCAO group (Figure 2). The pathological changes in the hippocampal tissues of the rats were relieved effectively in the miR-1 inhibitor group but aggravated distinctly in the miR-1 mimic group.

### 3.4. Changes in mRNA Expressions of miR-1, ERK1/2, Bcl-2, and Bax in Brain Tissues in each Group of Rats

According to Figure 3, compared with the sham group, the mRNA expression of miR-1 and Bax in the brain of model rats increased significantly (*p* < 0.05), and the mRNA expression of ERK1/2 decreased significantly. Compared with the model group, the mRNA expression of miR-1 and Bax in the brain tissues of rats in the miR-1 inhibitor group was significantly decreased, and the mRNA expression of ERK1/2 and Bcl-2 was significantly increased. The mRNA expression of miR-1 and Bax was significantly decreased, and the mRNA expression of Bcl-2 was significantly increased (*p* < 0.05) in the brain of rats in the miR-1 mimic group.

### 3.5. Comparison of Cranial Nerve Cell Apoptosis among Groups

The MCAO group and miR-1 mimic group had enhanced nerve cell apoptosis in the brain tissues compared with the sham group, but the miR-1 inhibitor group exhibited no apparent changes in nerve cell apoptosis in the brain tissues (Figure 4). Moreover, in comparison with the MCAO group, the miR-1 inhibitor group displayed weakened nerve cell apoptosis in the brain tissues, while the miR-1 mimic group showed no obvious changes in nerve cell apoptosis.

### 3.6. Protein Expressions of ERK, Bcl-2, Bax, and Caspase-3 in Brain Tissues in each Group of Rats

As shown in Figure 5, compared with the sham group, the protein of ERK1/2 in the model group decreased significantly, the protein of Bcl-2, Bax, and caspase-3 increased significantly, and the protein of ERK1/2, Bcl-2, Bax, and caspase-3 increased significantly in the miR-1 inhibitor group and the miR-1 mimic group; Compared with the model group, the protein levels of ERK1/2 and Bcl-2 in the miR-1 inhibitor group were significantly increased, the proteins of Bax and caspase-3 were significantly decreased, and the protein levels of ERK1/2 and Bcl-2 in the miR-1 inhibitor group were significantly increased (*p* < 0.05). Figure 5 shows the ERK, Bcl-2, Bax, and caspase-3 protein expressions in the brain of rats in each group.

RETRACTED

## 4. Discussion

In China, cerebral stroke is the leading cause of disability in adults, and it is the second major cause of death in people aged over 60 years old [11]. In addition, cerebral stroke is the fifth most important cause of death in population aged 15-59 years old in the world. About 2.4 million cases of cerebral stroke events have been recorded since 2013; 75% of which suffer from different degrees of disability [12]. It has been revealed in studies that cell apoptosis is a crucial reason of nerve cell death triggered by cerebral I/R injury [13–15]. The mitogen-activated protein kinase (MAPK)/ERK signaling pathway participates in the regulation of such biological processes as cell proliferation, differentiation, and apoptosis through modulating the activity of transcription factors. Moreover, the abnormal activation of the MAPK/ERK signaling pathway can induce cell apoptosis [16].

As a category of conserved small noncoding RNAs, miRNAs can repress protein translation at the posttranscriptional level via complementary base pairing with the specific 3′-UTR of mRNAs, so the abnormal expression of miRNAs is closely associated with various diseases [17]. Studies have demonstrated that aberrant miR-1 expression will affect the occurrence and development of diverse diseases. It is also investigated that miRNAs are capable of degrading the mRNAs of target genes and inhibiting their translation, thus playing vital roles in regulating pathophysiological processes such as cell proliferation, differentiation, and apoptosis [18–20]. miR-1 is currently known to be mainly expressed in the skeletal muscle and myocardium, and it is involved in the modulation of heart development, arrhythmia, myocardial ischemia, and other pathological processes according to studies [21]. It can be seen that miR-1 has close correlations with multiple diseases.

In this research, modified MCAO method was applied to establish the rat model of cerebral I/R injury, and miR-1 mimic and miR-1 inhibitor were utilized to investigate the impacts of ERK on the nerve cell apoptosis in rats with cerebral stroke. Then, the rats were administered with miR-1 inhibitor and miR-1 mimic for 3 consecutive days after successful modeling, and the cerebral infarction area and volume in the brain tissues of the rats were measured via TTC staining. It was found that there were fairly apparent infarcted tissues in the MCAO group, while the infarction area and volume were decreased remarkably after inhibiting miR-1, suggesting that the suppression of miR-1 can ameliorate the infarction caused by I/R injury in the rats. Later, the HE staining was performed to observe the hippocampal tissues in the rat brain, and it was discovered that the infarction in the rats was relieved after inhibiting miR-1. According to studies, miR-1 can affect cardiomyocyte apoptosis by influencing the ERK signaling pathway. Therefore, the mRNA expression of ERK1/2 in the brain tissues of rats was detected via qRT-PCR, and the results manifested that miR-1 was able to influence the ERK expression in the brain tissues of rats. Subsequently, the nerve cell apoptosis in the brain tissues of rats was determined by means of flow cytometry, and it was shown that repressed miR-1 could improve the nerve cell apoptosis in the brain tissues of rats with I/R injury. In contrast, miR-1 mimic could enhance the nerve cell apoptosis in rats, illustrating that miR-1 can intervene in the nerve cell apoptosis in rats through ERK. Finally, the above conclusions were verified using Western blotting.

RETRACTED

Nevertheless, the precise mechanism of miR-1 in affecting the nerve cell apoptosis in rats with cerebral stroke may also be related to other target genes of miR-1. A latest study indicated that the level of miR-1 rises in cardiomyocytes, and the overexpression of miR-1 attenuates the phosphorylation of MAPK and the activation of PI3K p85*α* and regulates the energy metabolism of cardiomyocytes by virtue of IRS2, Akt, and ERK. It has been revealed that miR-1 regulates diversified target genes, including MTSS1, HOXA10, SMAD5, and JAK2. In this research, however, the impacts on the ERK signaling pathway were merely testified, while the impacts on other signaling pathways were not elaborated, which will lay an experimental foundation for subsequent studies on the pathogenesis of nerve cell apoptosis in rats with cerebral stroke.

## Figures and Tables

**Figure 1:** TTC staining results of brain tissues in each group. Note: (a) sham-operation group, (b) MCAO: model group, (c) miR-1 inhibitor group, and (d) miR-1 mimic group.

**Figure 2:** Pathological changes in hippocampal tissues in each group of rats (HE staining, ×200). Note: (a) sham-operation group, (b) MCAO: model group, (c) miR-1 inhibitor group, and (d) miR-1 mimic group.

**Figure 3:** mRNA expression of miR-1, ERK1/2, Bcl-2, and Bax in the brain of rats from each group. Note: sham: sham-operation group; MCAO: model group; miR-1 inhibitor: miR-1 inhibitor group; miR-1 mimic: miR-1 mimic group, ^∗^*p* < 0.05 and ^∗∗^*p* < 0.01 vs. the sham group.

RETRACTED

**Figure 4:** Influence on cranial nerve cell apoptosis in each group of rats. Note: (a) sham-operation group, (b) MCAO: model group, (c) miR-1 inhibitor group, and (d) miR-1 mimic group.

**Figure 5:** Protein expressions of ERK, Bcl-2, Bax, and caspase-3 in brain tissues in each group of rats. (a) Western blot result. (b) Quantification analysis. ^a^*p* < 0.05 vs. the Sham group, ^b^*p* < 0.05 vs. the MCAO group. Note: sham: sham-operation group; MCAO: model group; miR-1 inhibitor: miR-1 inhibitor group; miR-1 mimic: miR-1 mimic group.

**Table 1:** EZ Longa scoring criteria.

No.	Symptom	Score
1	There is not any symptom of neurological deficit.	0
2	The right forepaw cannot straighten completely.	1
3	The rat tilts to the right involuntarily or circles to the right when walking.	2
4	The rat tumbles to the right or has paralysis of the right side of the body when walking.	3
5	The rat has coma and cannot walk autonomously.	4
6	The rat dies.	5

**Table 2:** Primer sequences for qRT-PCR.

Primer	Sequence
miR-1	5′-CGTCCTTCAAGTAATCCAGGA-3′
	5′-GCAGGGTCCGAGGTATTC-3′
ERK1/2	5′-GAACTCCAAGGGCTATACCAAGT-3′
	5′-GGAGGGCAGAGACTGTAGGTAGT-3′
B-cell lymphoma-2 (Bcl-2)	5′-CCGGGAGATCGTGATGAAGT-3′
	5′-ATCCCAGCCTCCGTTATCCT-3′
Bcl-2-associated X protein (Bax)	5′-GTGGTTGCCCTCTTCTACTTTG-3′
	5′-CACAAAGATGGTCACTGTCTGC-3′
GAPDH	5′-AGGTCGGTGTGAACGGATTTG-3′
	5′-TGTAGACCATGTAGTTGAGGTCA-3′

**Table 3:** Comparison of neurological deficit after MCAO among groups (points, $\bar{\chi }\pm s$).

Group	*n*	Neurological deficit score
Sham group	10	0.31 ± 0.07
MCAO group	10	2.49 ± 0.55^a^
miR-1 inhibitor group	10	0.79 ± 0.27^b^
miR-1 mimic group	10	3.65 ± 0.52^ab^

^a^*p* < 0.05 vs. the Sham group, ^b^*p* < 0.05 vs. the MCAO group.

**Table 4:** Comparison of cerebral infarction volume after MCAO among groups ($\bar{\chi }\pm s$).

Group	*n*	Cerebral infarction volume (%)
Sham-operation group	10	1.08 ± 0.05
MCAO group	10	42.48 ± 8.42^a^
miR-1 inhibitor group	10	16.18 ± 3.45^b^
miR-1 mimic group	10	50.44 ± 5.58^a^

^a^*p* < 0.05 vs. the Sham group, ^b^*p* < 0.05 vs. the MCAO group.

## Data Availability

The datasets used and/or analyzed during the current study are available from the corresponding author on reasonable request.
